The article "Amelioration of obsessive-compulsive disorder in three mouse models treated with one epigenetic drug: unraveling the underlying mechanism" was retracted in 2021. Reasons: errors in the materials; errors in the results or conclusions; duplicate publication; unreliable results or conclusions.

# Amelioration of obsessive-compulsive disorder in three mouse models treated with one epigenetic drug: unraveling the underlying mechanism

**DOI:** 10.1038/s41598-019-45325-6

**Published:** 2019-06-19

**Authors:** German Todorov, Karthikeyan Mayilvahanan, David Ashurov, Catarina Cunha

**Affiliations:** 1 Emotional Brain Institute, Nathan Kline Institute, Orangeburg, NY USA; 2 Department of Neurobiology and Behavior, Stony Brook University School of Medicine, Stony Brook, NY USA

**Keywords:** Obsessive compulsive disorder, Epigenetics and behaviour, Habituation

## Abstract

Mental health disorders are manifested in families, yet cannot be fully explained by classical Mendelian genetics. Changes in gene expression via epigenetics present a plausible mechanism. Anxiety often leads to avoidant behaviors which upon repetition may become habitual, maladaptive and resistant to extinction as observed in obsessive compulsive disorders (OCD). Psychophysical models of OCD propose that anxiety (amygdala) and habits (dorsolateral striatum, DLS) may be causally linked. The amygdala activates spiny projection neurons in the DLS. Repetitive amygdala terminal stimulation in the DLS elicits long term OCD-like behavior in mice associated with circuitry changes and gene methylation-mediated decrease in the activity of protein phosphatase 1 (PP1). Treatment of OCD-like grooming behavior in Slitrk5, SAPAP3, and laser-stimulated mice with one dose of RG108 (DNA methyltransferase inhibitor), lead to marked symptom improvement lasting for at least one week as well as complete reversal of anomalous changes in circuitry and *PP1* gene methylation.

## Introduction

Mental health disorders repeatedly arise in families and often co-occur in twins, but most cases cannot be explained by classical Mendelian genetics. The current model, which could help solve this conundrum, involves long-term modifications in gene expression that are influenced by environmental factors and sometimes are passed onto the following generations (epigenetics)^1^. Novel studies propose that modulations in gene expression influenced by environmental factors, are connected to mental health disorders^2–14^.

Epigenetic mechanisms^15,16^ are essential for normal development and cell differentiation as a way to generate and maintain different specialized tissue-specific phenotypes based on the same genome^17^. There is accumulating evidence that epigenetic mechanisms have been re-purposed in the nervous system as regulatory participants in long-term neuronal changes essential for neuroplasticity, learning, long-term memory and related functions^18–21^. DNA methylation is a key epigenetic mechanism that most commonly involves covalent modification of DNA at 5′ position of cytosine (5mC) by the class of enzymes called DNA methyltransferases (DNMT), which could induce long-term gene expression changes (usually silencing but occasionally activation, depending on the region) by preventing RNA-polymerase and transcription factor binding. In mammals, 5mC is highly prevalent and occurs most commonly but not exclusively in CpG pairs^22,23^.

The article "Amelioration of obsessive-compulsive disorder in three mouse models treated with one epigenetic drug: unraveling the underlying mechanism" was retracted in 2021. Reasons: errors in the materials; errors in the results or conclusions; duplicate publication; unreliable results or conclusions.

Non-CpG methylations (CpA, CpT and CpC) also occur but appear to be largely restricted to a few specific cell types, notably neurons and glial cells^22,24,25^.

There is also evidence of DNA methylation at N6 position of adenine in both prokaryotes and eukaryotes^26^. However, in mammals, the levels of N6-adenine DNA methylation appear to be very low, except during embryogenesis^26^, and its physiological role is poorly understood^27^. N6-adenine DNA methylation does not appear to have any proven regulatory role in the adult mammalian cells^28,29^. The mammalian enzymes responsible for N6-adenine DNA methylation have not been conclusively identified.

DNMTs are generally expressed and active during development, cell division, and differentiation. They play a major role in setting transcriptional patterns for the differentiated phenotype, which then remain stable over the lifespan of cells. It was believed that once a methylation pattern is set by DNMTs, it remained static in differentiated cells. However, mammalian adult nervous system has comparatively high DNMT activity^30,31^. The DNMT enzyme family has a number of subtypes that appear to be functionally different. In mammals, subtypes include DNMT1, DNMT2 (a.k.a. TRDMT1), DNMT3A and DNMT3B. In terminally differentiated neurons in adult brains, DNMT1, DNMT3A and DNMT3B appear to be active and possibly dynamically regulated. Studies show that DNMT activity is necessary for long-term memory formation and that DNMT inhibition disrupts long-term memory^21^. DNMT3A appears to be the specific subtype required for normal *de novo* learning and memory. Forebrain specific DNMT3A knockout mice, but not DNMT1 knockout mice, exhibited altered LTP and synaptic plasticity in the affected areas as well as learning and memory deficits^32^. On the other hand, it appears that both DNMT1 and DNMT3A are required for maintenance of methylation and synaptic function as indicated by double-knockout studies^33^.

In our study we focused on obsessive compulsive disorders (OCD). To assess the role of DNA methylation in OCD-like behaviors, we used two genetic mouse models of OCD-like grooming behavior: SAPAP3 and Slitrk5 knockout (KO) mice^34,35^. Both SAPAP3 and Sltirk5 KO mice, which exhibit a high degree of OCD-like grooming behavior and anxiety-like behaviors, are considered relevant models for the corresponding human conditions, such as OCD. In fact, mutations in Sltirk5 and SAPAP3 have been linked to increased risk of OCD in humans^36,37^.

The article "Amelioration of obsessive-compulsive disorder in three mouse models treated with one epigenetic drug: unraveling the underlying mechanism" was retracted in 2021. Reasons: errors in the materials; errors in the results or conclusions; duplicate publication; unreliable results or conclusions.

SAPAP3 KO mice lack one of SAP90/PSD-95-associated proteins (SAPAPs, also known as guanilate cyclase associated proteins), a family of scaffold proteins in postsynaptic density^34^. The net effect of deleting SAPAP3 appears to be the reduction of the sensitivity to AMPAR-mediated glutamatergic signaling.

Slitrk5 KO mice lack a member of the Slitrk family encoding type 1 transmembrane proteins that localize at neuronal synapses and mediate synaptic formation and function through trans-synaptic interactions with presynaptic binding partners. Of the Slitr family, Slitr5 is particularly specific to striatum. The net effect of deleting Slitrk5 in striatum appears to be the reduction in sensitivity to neurotrophic signaling^38^.

Our third OCD mouse model uses optogenetic laser neuromodulation and is based on psychophysiological model of OCD-like behaviors, which proposes that anxiety (mediated by the amygdala) and habits (managed primarily by dorsolateral striatum or DLS) may be causally linked^39^. The DLS is composed of two types of spiny projection neurons (SPNs) that project to different targets, receive different excitatory inputs and respond differently to neuromodulators. The so-called indirect pathway SPNs (iSPNs) express D2 type dopamine receptors and ultimately suppress movement by inhibiting thalamic output, while D1 receptor expressing direct pathway neurons (dSPNs) promote it. We have recently shown that the basal and lateral nuclei of the amygdala (BLA) send functional projections directly to SPNs in the DLS, and that these projections target D1s and D2s similarly in wild type (WT) mice^40^. Furthermore, repeated activation of the BLA-DLS pathway promoted the generation of long-lasting OCD-like grooming behavior^41^. We treated the OCD-like behavior in the 3 mice models, by subcutaneously injecting a single dose of an epigenetic drug RG108, a non-nucleoside DNA methyltransferase (DNMT) inhibitor. The drug effectively reduced OCD-like behavior in all 3 mice models. In the WT laser-stimulated mice we showed that drug application before laser stimulation prevented the induction of OCD-like behavior. Open field and elevated plus maze test showed that anxiety levels were similar to unstimulated WT mice. We found that circuitry alterations in the RG108 treated mice were back to baseline levels comparable to non-stimulated WT mice. Using qPCR, we examined the role of DNMT methylation in memory, and looked for direct evidence of altered DNA methylation. Protein phosphatase 1 (PP1) is a memory formation inhibitor, and *PP1* gene methylation was shown to regulate its expression and activity^21,42^. We observed a marked increase in methylation level of *PP1* gene in the laser-stimulated left hemisphere compared to the unstimulated right hemisphere of the DLS. The increase in *PP1* methylation was completely reversed by RG108 injection. These results support the hypothesis that mental health disorders may arise, at least in some cases, from epigenetic modulations leading to impairments of cellular plasticity cascades, which induce aberrant information processing in the circuits. Future disorder-specific, effective and potentially curative therapies would require inducing targeted neuronal plasticity changes to help restore appropriate synaptic function and neuronal connectivity. This study may have implications not only for OCD but also for a variety of complex disorders such as Parkinson’s, schizophrenia, autism, anxiety, and addiction, where the circuits overlapping or resembling the ones we studied have been implicated^43^.

The article "Amelioration of obsessive-compulsive disorder in three mouse models treated with one epigenetic drug: unraveling the underlying mechanism" was retracted in 2021. Reasons: errors in the materials; errors in the results or conclusions; duplicate publication; unreliable results or conclusions.

## Results

### Epigenetic modulator drugs reduce OCD-like behavior in two different genetic mouse models of OCD

We injected subcutaneously a single dose of RG108, a non-nucleoside DNA methyltransferase (DNMT) inhibitor, in two different genetic mouse models of OCD-like over grooming behavior Slitrk5-deficient and SAPAP3-deficient mice^34,35^, which reduced this behavior significantly (p < 0.05, Fig. 1a). In Slitrk5-deficient mice the effect of the drug was long-lasting and led to reduction of over-grooming-inflicted lesions, while in the SAPAP3-deficient mice the effect only persisted for 3 days (Fig. 1a). SAPAP3-deficient mice seem to represent a more persistent case of OCD-like grooming behavior partially resistant to long lasting epigenetic modulatory effects of RG108. In the next set of experiments, we administered subcutaneously sodium butyrate (NaB), which inhibits class I histone deacetylase (HDAC) activity, inducing histone hyper-acetylation,^44,45^, and was shown to strengthen cocaine-associated contextual memory^46^. We observed that in the SAPAP3-deficient and Slitrk5-deficient mice the OCD-like grooming behavior was increased in all mice (p < 0.05). A single injection of RG108 reduced the OCD-like grooming behavior immediately in all mice and was long lasting (at least 7 days) in Slitrk5-deficient mice (p < 0.05, Fig. 1b).

**Figure 1:** RG108 effectively reduced and prevented maladaptive habitual avoidance-like behavior in two different genetic mouse models. (**a**) Single subcutaneous injection of RG108 into Slitrk5 KO (more than 7 days) and SAPAP3 KO (3 days) mice reduced habitual grooming behavior. N = 5–6; p < 0.05 KO saline group is a mix of both KOs (N = 4 and N = 4). (**b**) Single subcutaneous injection of sodium butyrate (NAB) into Slitrk5 KO and SAPAP3 KO mice increased habitual grooming behavior. N = 5–6; p < 0.05. Injection of RG108 after NAB application reversed the increased habitual grooming behavior. N = 5–6; p < 0.05.

The article "Amelioration of obsessive-compulsive disorder in three mouse models treated with one epigenetic drug: unraveling the underlying mechanism" was retracted in 2021. Reasons: errors in the materials; errors in the results or conclusions; duplicate publication; unreliable results or conclusions.

### *PP1* gene methylation levels are proportionate to OCD-like behavior levels in KO mice

To gain a deeper insight into the role of RG108 in OCD-like behavior, we tested for direct evidence of altered DNA methylation related to memory. Studies of contextual fear conditioning and novel object recognition suggest that protein phosphatase 1 (*PP1*) is a memory suppressor gene^21,42^. The inhibition of *PP1* activity enhances LTP, the efficacy of associative training, and the maintenance of memory^42,47,48^. Analysis of *PP1* expression patterns in the mammalian brain demonstrates that *PP1* is most abundantly expressed in the striatum^49^ and that *PP1* expression and activity are regulated by its methylation state^21,42^. We performed methylation-specific quantitative real-time PCR to examine methylation changes in the DLS of the specific target gene *PP1* in the different mouse models of OCD with and without drug application. We detected the levels of methylated *PP1* of 5.2 log-2-fold-change in untreated KO mice relative to WT controls (p < 0.01, Fig. 2). Treatment with RG108 reduced the level of methylated *PP1* to an undetectable level while the level of un-methylated *PP1* increased to an over 4.02 log-2-fold-change (p < 0.01, Fig. 2). NaB injection downregulated the level of un-methylated *PP1*, resulting in −5.5 log-2-fold-change, and increased the level of methylated *PP1, leading* to an 13.86 log-2-fold-change (p < 0.01, Fig. 2).

**Figure 2:** *PP1* gene methylation in KO mice. *PP1* methylated and un-methylated levels (comparison to WT mice) of untreated vs RG108 and NAB treated KO mice. N = 4. p < 0.05.

Considering both the behavior and gene methylation results, we concluded, that our BLA-DLS pathway laser-stimulated WT mice might represent a valid and useful mouse model for OCD-like behavior. Additionally, this mouse model allowed us to control neuromodulation precisely (time point, duration, localization, intensity, and frequency), which would enable us to gain deeper insights into underlying mechanisms of OCD-like behavior. Therefore, we wanted to study further which underlying mechanisms took place in laser-stimulated WT mice showing OCD-like behavior. The inhibitory mechanism of RG108 appears to be direct and specific, and it shows comparatively low toxicity in human cancer cell lines^50^. This makes RG108 is an interesting candidate for further studies as a potential therapeutic agent. Therefore, we will focus our next experiments on RG108.

The article "Amelioration of obsessive-compulsive disorder in three mouse models treated with one epigenetic drug: unraveling the underlying mechanism" was retracted in 2021. Reasons: errors in the materials; errors in the results or conclusions; duplicate publication; unreliable results or conclusions.

### Epigenetic modulator RG108 reduces OCD-like behavior in optogenetic laser neuromodulation mouse model of OCD

Our third mouse model for OCD-like behavior is based on optogenetic laser neuromodulation (Fig. 3).

**Figure 3:** *In vivo* optogenetic activation of BLA inputs to the dorsolateral striatum. (**a**) Injection of AAV-synapsin-ChR2-GFP construct into the basal and lateral amygdala (BLA). Placement of fiberoptic cannulas and blue laser stimulation in DLS. The dorsolateral striatum was stimulated by a blue laser coupled to an implanted cannula for 10 minutes a day, over 5 days, in mice receiving AAV-ChR2 or saline injections into the BLA. (**b**) Example injection site of AAV-synapsin-ChR2-GFP construct into the BLA. **c** Example placement of fiberoptic cannula in DLS.

The previously described knock out mice present a genetic mouse model of OCD. However, most cases of mental health disorders cannot be fully explained by classical Mendelian genetics. Based on that knowledge, we wanted to study which brain circuitry modulations could represent an underlying or contributing mechanism for OCD. Psychophysical models of OCD propose that anxiety (represented by the amygdala) and habits (involvement of the DLS) may be causally linked^39^. We recently showed that the BLA sends functional projections directly to striatal spiny projection neurons (SPNs) in the dorsolateral striatum (DLS), and that these projections target direct pathway SPNs (D1s) and indirect pathway SPNs (D2s) similarly in WT mice^40^. Repeated optogenetic *in vivo* stimulation of BLA axon terminals in the DLS gradually induced long lasting OCD-like grooming behavior in WT mice (p < 0.05, Fig. 4a). We injected one dose of RG108, into the laser-stimulated mice which lead to a reversal of OCD-like grooming behavior lasting for at least one week (p < 0.05, Fig. 4a). In order to study if RG108 was able to prevent OCD-like grooming behavior, we injected the drug 10 min before each laser stimulation session, which confirmed our hypothesis (p < 0.05, Fig. 4b).

**Figure 4:** RG108 effectively reduced and prevented OCD-like (over grooming) behavior in laser stimulated WT mice. (**a**) Unilateral stimulation of the BLA input in the dorsolateral striatum with a blue laser coupled to an implanted cannula for 10 minutes a day, over 5 days, in mice receiving RG108 or saline injections 10 min before laser stimulation. The second control group had implanted sham cannulas, so the laser stimulation didn’t show an effect on grooming behavior. **Behavior was measured for 5 min before daily laser stimulation, as well as 3 and 7 days after last stimulation**. N = 5–7; p < 0.05. (**b**) The dorsolateral striatum was stimulated by a blue laser coupled to an implanted cannula for 10 minutes a day, over 5 days, in mice. After 3 days of the last laser stimulation the mice received RG108 or saline injections. Behavior was measured for 5 min before daily laser stimulation. Unilateral activation of BLA inputs increased OCD-like behavior (over grooming). After RG108 injection the OCD-like behavior was reduced. Saline injections didn’t have this effect. N = 5–7; p < 0.05.

The article "Amelioration of obsessive-compulsive disorder in three mouse models treated with one epigenetic drug: unraveling the underlying mechanism" was retracted in 2021. Reasons: errors in the materials; errors in the results or conclusions; duplicate publication; unreliable results or conclusions.

### *PP1* gene methylation levels are proportionate to modulated OCD-like behavior levels in laser-stimulated WT mice

We studied *PP1* methylation state (levels of methylated and un-methylated forms of *PP1*) in the optogenetic laser neuromodulation (unilateral left hemisphere) mouse model of OCD with and without drug application in the DLS. We found the levels of un-methylated *PP1* to be higher in the right hemisphere DLS (3.8 log-2-fold-change) than in the stimulated left hemisphere DLS (1.8 log-2-fold-change, p < 0.01, Fig. 5). The opposite was detected for the methylated *PP1* levels, where the right hemisphere showed low levels of a 1.2 log-2-fold-change and the left hemisphere had high levels of 8.7 log-2-fold-change (p < 0.01, Fig. 5). A single injection of RG108 significantly downregulated methylated *PP1* levels to negative values (below control baseline) in both hemispheres, with −3.5 and −3.7 log-2-fold-change in the right and left DLS correspondingly (p < 0.01, Fig. 5).

**Figure 5:** *PP1* gene methylation in WT mice. Comparison (to WT unstimulated) of *PP1* methylated and un-methylated levels of WT unilateral (left hemisphere) laser stimulated untreated mice and RG108 treated right vs left hemisphere. N = 4 p < 0.05.

### RG108 modulates anxiety-like behavior

Laser-stimulated WT mice spent significantly less time in the center of the open field than sham cannula mice (p < 0.05). Laser-stimulated mice that were injected with a single dose of RG108 spent as much time in the center of the open field as the sham cannula mice. Elevated plus maze tests showed that untreated laser-stimulated WT mice spend the least time in open arms compared to RG108 treated laser-stimulated WT mice and laser-stimulated WT mice implanted with sham cannulas (Fig. 6a,b, p < 0.05).

**Figure 6:** RG108 reduced anxiety-like behavior. (**a**) Time spent in the center of open field was significantly different between laser stimulated and sham cannula mice. RG108 injection increased the time spent in the open field of laser-stimulated mice. N = 5; p < 0.05. (**b**) The mobility measured by distance traveled during the open field test is not different between groups. N = 5; p > 0.05. (**c**) RG108 injected mice showed similar behavior in the elevated plus maze as the control mice. N = 5; p < 0.05.

The article "Amelioration of obsessive-compulsive disorder in three mouse models treated with one epigenetic drug: unraveling the underlying mechanism" was retracted in 2021. Reasons: errors in the materials; errors in the results or conclusions; duplicate publication; unreliable results or conclusions.

### Circuitry alterations induced by laser stimulation of the BLA-DLS pathway were reversed in RG108 treated mice, and comparable to non-stimulated WT mice

In order to measure paired pulse ratios (PPR), we used acute coronal brain slices where we stimulated with 2 laser pulses (1 μm radius) the same spot using a 100 ms interval, the BLA input onto the SPNs in the DLS 400 um away from recorded neurons. We observed paired pulse depression (PPD) in the BLA input to the SPNs of the DLS in WT mice. In brain slices from *in vivo* laser-stimulated WT mice showing OCD-like behavior, we recorded a reduction in PPRs in D1s of the DLS (Fig. 7a,b, p < 0.05). Injection of RG108 reversed this effect in the D1s (Fig. 7a,b, p < 0.05).

**Figure 7:** Circuitry alterations of the RG108 treated mice were back to baseline levels comparable to non-stimulated WT mice. (**a**) PPR evaluated at 100-millisecond (msec) intervals. The PPR values were computed as the ratio of the second stimulus-evoked EPSC peak divided by the first stimulus-evoked EPSC peak. The PPRs of WT and laser stimulated WT DLS slices (WT saline: D1 N = 8, D2 N = 7; WT laser stimulated: D1 N = 8, D2 N = 7, RG108 injected D1 N = 8, D2 N = 9) were calculated from the averaged PPR values. p < 0.05. (**b**) Example traces of D1 recordings under control conditions, after laser stimulation and application of RG108. N = 9 D1s. (**c**) Relative NMDA/AMPA receptor contribution is elevated at BLA-D1 synapses in laser stimulated mice, and RG108 injection reverses the levels back comparable to controls. EPSCs evoked by full-field optogenetic stimulation in mice receiving stereotaxic ChR2 injections into BLA or sensorimotor cortex; NMDA/AMPA receptor-mediated synaptic contributions measured. N = 9 D1s and N = 9 D2s; p < 0.05. d Example traces of dSPN recordings under control conditions, after laser stimulation and application of RG108. N = 9 D1s.

In order to detect changes in NMDA/AMPA ratios, we recorded in voltage clamped SPNs BLA input laser stimulation evoked AMPA currents at −70 mV, and NMDA currents at +40 mV. D1s in the DLS from laser-stimulated WT mice displaying OCD-like behavior, showed a significant increase in NMDA/AMPA ratios, which was reversed through RG108 treatment (Fig. 7c,d, p < 0.05).

High magnification images (5 × Zoom) of SPN dendrites in the DLS showed a higher spine density in D1s in laser-stimulated mice with OCD-like behavior compared to controls (sham cannula). RG108 reversed this effect and re-established the balance between the direct and indirect pathway (Fig. 8a,b, p < 0.05).

The article "Amelioration of obsessive-compulsive disorder in three mouse models treated with one epigenetic drug: unraveling the underlying mechanism" was retracted in 2021. Reasons: errors in the materials; errors in the results or conclusions; duplicate publication; unreliable results or conclusions.

**Figure 8:** Repeated *in vivo* stimulation of BLA inputs to the dorsolateral striatum increases WT spine density mainly in the D1s and RG108 reverses it. (**a**) Measurements taken a week after the last stimulation and drug injection. Drug manipulation recapitulates the same spine density seen in unstimulated (sham) WT mice. N = 9–16. p < 0.05. (**b**) Example dendritic spines under different conditions.

## Discussion

Our results show that a single dose of DNMT inhibitor RG108 markedly reduced maladaptive habitual grooming behavior in both SAPAP3 and Sltirk5 KO mice. In Slitrk5 KO mice, grooming **decreased** to the normal level and remained within the wild type (WT) range for at least 7 days after the treatment. In SAPAP3 KO mice, whose pathological habitual grooming is more severe compared to Slitrk5, over-grooming decreased markedly but was still above the WT range. The behavior improvement in SAPAP3 KO mice lasted between 3 and 7 days’ post-treatment–on day 7 post-treatment, the over grooming was only mildly below the pre-treatment level.

**Furthermore,** we found that a single dose of HDAC inhibitor sodium butyrate (NaB) markedly increased OCD-like behavior (over-grooming) in both in SAPAP3 and Sltirk5 KO mice, the effect being especially dramatic in SAPAP3 mice. In both KO mouse strains, the over-grooming increase was the greatest 30 minutes after the injection, gradually decreasing over the next few days and still above the original baseline on day 7. The stimulatory effect of HDAC inhibitor NaB on over-grooming in KO mice was completely offset by concurrent administration of DNMT inhibitor RG108, the resultant grooming level dropping below the original baseline. Thus DNMT inhibitor not only partially or completely suppressed pathological OCD-like behavior in KO mice but also overcame the opposing stimulatory effect of HDAC inhibition.

To further verify the role of epigenetic mechanisms in the observed effects and to identify a potential regulatory target we used qPCR to analyze methylation levels of protein phosphatase 1 (*PP1*) gene in KO mice. PP1 inhibits memory formation and learning^42^. Since habit formation in OCD-like behavior can be viewed as a variant of the memory/learning mechanism, we presumed *PP1* to be among the likely regulators involved. Furthermore, previous studies reported that an increase in *PP1* methylation reduced its expression, which lead to a decrease in memory inhibition^21^.

We found that DNMT inhibition lead to a marked reduction in *PP1* methylation in the DLS of the KO mice. Conversely, HDAC inhibition lead to changes in the opposing direction: a marked increase in *PP1* methylation and presumably the corresponding reduction in the *PP1* expression^21^.

The article "Amelioration of obsessive-compulsive disorder in three mouse models treated with one epigenetic drug: unraveling the underlying mechanism" was retracted in 2021. Reasons: errors in the materials; errors in the results or conclusions; duplicate publication; unreliable results or conclusions.

HDAC is known to enhance memory and synaptic plasticity via CREB:CBP-dependent signally^51^. Additionally, a recent study reported that suppression of HDAC3 function in DLS accelerates habit formation whereas HDAC3 overexpression prevents it^52^. HDAC3 is a class I HDAC highly expressed in the brain and believed to be enriched at learning-related and CREB-regulated gene promoters^53,54^. Conversely, the CREB phosphorylation by PP1 was reported to suppress CREB activity^55^. In that context, our data on the opposing effects of DNMT and HDAC inhibition on maladaptive habitual behaviors and *PP1* activity suggest the opposing effects of DNA demethylation and histone acetylation on CREB:CBP-dependent pathway, which is known to be involved in neuroplasticity^56,57^. In fact, PP1 and CREB:CBP may represent a key nexus of epigenetic regulation of neuroplasticity occurring during the development and reversal of OCD-like behaviors.

At present, SAPAP3 and Sltirk5 KO mice are arguably the most clinically relevant models of OCD-like behaviors available in rodents. Yet it remains unclear how these genetic lesions lead to the behavioral manifestations, which makes interpreting the effects of epigenetic interventions in the KO mice more difficult. Slitrk5 deletion was shown to reduce the sensitivity to neurotrophic signaling by BDNF^35^ whereas SAPAP3 deletion appears to reduce the sensitivity to AMPAR-dependent glutamatergic signaling^34^. A long-term reduction in DLS sensitivity to inputs, whether via BDNF or AMPA pathway, would likely produce compensatory regulatory changes in the DLS and, perhaps more importantly, in the circuits connected to it from BLA, thalamus and cortex. Such compensatory changes may favor inputs via movement stimulating dSPN circuitry over the inhibitory iSPN circuitry, facilitating excessive LTP and more sustained upstates in dSPNs in the DLS, thus lowering the trigger threshold of OCD-like behaviors. This hypothesis is consistent with our findings but requires substantial further investigation to confirm.

Why is the suppression of over-grooming by DNMT inhibition less sustained in SAPAP3 KO mice? SAPAP3 KO mice show much more severe over-grooming than Sltirk5 KO or BLA-DLS laser-stimulated WT mice. This may reflect a far greater level of baseline imbalance between movement activating (D1) and inhibitory (D2) pathway in DLS circuitry. A highly intense and sustained activation is known to cause not only transient synaptic changes but also a longer-term one (LTP, LTD), partly via epigenetic modifications^58^. Hence it is possible that in the case of SAPAP3 KO mice, epigenetic changes produced by a single dose of DNMT inhibitor are more likely to be reversed over time.

The article "Amelioration of obsessive-compulsive disorder in three mouse models treated with one epigenetic drug: unraveling the underlying mechanism" was retracted in 2021. Reasons: errors in the materials; errors in the results or conclusions; duplicate publication; unreliable results or conclusions.

We found that in WT mice DNMT inhibition caused a dramatic, rapid, and sustained improvement in OCD-like behaviors induced by laser stimulation. A single RG108 injection suppressed over-grooming in laser-stimulated mice for at least seven days. A similar improvement was observed in anxiety-like behavior in elevated plus maze. We showed that behavioral changes associated with laser stimulation and RG108 injection correlated with changes in circuitry. Additionally, laser stimulation of BLA-DLS inputs increased the density of D1 dendritic spines and produced changes in D1 & D2 paired pulse and AMPA/NMDA ratios, which correlated with the exacerbation of maladaptive behaviors. DNMT inhibition reversed laser stimulation-induced circuitry changes, such that BLA-DLS inputs resembled (functionally and morphologically) those in unstimulated WT mice. Laser stimulation-induced OCD-like behavior in WT mice was associated with an increase in *PP1* gene methylation in the DLS of the left hemisphere (unilateral stimulation) to levels comparable to those in KO mice. Conversely, only mild *PP1* methylation changes were observed in the right hemisphere (contralateral side of unilateral stimulation). A single treatment of the laser-stimulated WT mice with DNMT inhibitor RG108 completely reversed *PP1* methylation increase in the DLS.

The high degree of alignment between observed behavioral and regulatory effects of epigenetic modulation in both gene knockout and laser stimulation based mouse models point to the key physiological role of epigenetic mechanisms in OCD-like behaviors as well as likely clinical relevance of SAPAP3 and Stilrk5 KO mice as animal models. In fact, the aforementioned decrease in the striatum sensitivity to inputs and the resulting overcompensation/over activity of D1 movement stimulating circuit connections to DLS may not be limited to SAPAP3 and Stilrk5 KO mice. Numerous genetic and environmental factors may reduce striatum sensitivity and lead to maladaptive overcompensation, potentially accounting for a significant proportion of cases of pathological OCD-like behaviors.

Our results show that DNMT inhibition can trigger neuroplasticity and long-term synaptic changes in circuitry involved in OCD-like behaviors. Rapid onset of the behavioral changes we observed after DNMT inhibition indicates that the DNA methylation state of the affected neurons is not static. Inhibition of active methylation is likely to alter DNA methylation patterns (and thus gene expression and behavior) only if there is an active process of demethylation continuously opposing methylation in adult neurons. Since both DNMT and TET enzymes are continuously expressed in adult neurons^31,33,59^, they likely maintain a certain equilibrium level of methylation (dynamic steady state), which is apparently required in order to maintain the existing synaptic functions. Disrupting this methylation steady state by interfering with either DNMT (methylation) or TET (hydroxymethylation and demethylation) causes the opposing process to prevail, presumably by activating neuroplasticity/synaptic changes via CREB:CBP-dependent pathway. In our experiments, DNMT inhibition lead to rapid onset of behavioral changes presumably due to the decrease in methylation brought about by unopposed activity of TET enzymes. We can speculate that inhibition of DNMT1 and DNMT3A may be particularly important in the observed effects. Further studies targeting either specific DNMTs enzymes (via more specific inhibitors) or the expression of their genes (e.g. using miRNAs) in the context of OCD-like behaviors may help clarify the involvement of specific DNMT subtypes and suggest narrower therapeutic targets.

The article "Amelioration of obsessive-compulsive disorder in three mouse models treated with one epigenetic drug: unraveling the underlying mechanism" was retracted in 2021. Reasons: errors in the materials; errors in the results or conclusions; duplicate publication; unreliable results or conclusions.

Prior studies of TET activity in adult neurons suggest that the loss of methylation following DNMT inhibition is likely produced by an increase in hydroxymethylation by TET1 and/or TET3, subtypes shown to be involved in adult neuroplasticity^60^. Future research involving dynamic overexpression or repression of specific TET enzymes within striatum and related structures should clarify their role and therapeutic potential in obsessive-compulsive behaviors. Considering the potentiating effect of HDAC inhibition on OCD-like behaviors, investigating the effects of HDAC overexpression (especially HDAC3) and HAT inhibition may also yield new therapeutic targets.

Taken together, morphological (spine density), physiological (receptor and paired pulse ratios), and molecular (*PP1* gene methylation) changes associated with laser stimulation-induced OCD-like behavior in mice indicate long-term potentiation (LTP) in the BLA-DLS circuitry, specifically affecting D1s. We showed that all of the above changes are either completely reversed or markedly diminished by DNMT inhibition, indicating the sustained reversal of LTP, which could also be viewed as a form of long-term depression (LTD) of D1 BLA-DLS circuitry.

In fact, reduction in spine density is a common characteristic of LTD and involves limited synaptic apoptosis affecting spines^61^, which can be viewed as a form of synaptic pruning. Synaptic apoptosis/pruning appears to involve limited autophagy triggered via mTOR pathway by direct or indirect mTOR kinase inhibition. Modulation of mTOR pathway via epigenetic mechanisms involving DNA methylation and histone modifications was shown to play a role in memory reconsolidation^18^. It was found that memory retrieval was associated with transient suppression of mTOR pathway (activation of autophagy) while the subsequent reconsolidation was linked to mTOR pathway activation (suppression of autophagy), both involving epigenetic regulatory changes. These epigenetically mediated fluctuations in synaptic strength observed during memory retrieval and consolidation may have an equivalent in striatal activity involved in obsessive-compulsive behaviors. Activation of habitual motor behaviors is likely to rely on the same neuronal mechanisms as memory retrieval and reconsolidation and may also involve, even in a steady state, frequent epigenetically mediated fluctuation in synaptic strength. This would be consistent with our findings that epigenetic modulators can influence OCD-like behaviors. The role of synaptic apoptosis/pruning and mTOR pathway in OCD-like behavior should be further investigated.

The article "Amelioration of obsessive-compulsive disorder in three mouse models treated with one epigenetic drug: unraveling the underlying mechanism" was retracted in 2021. Reasons: errors in the materials; errors in the results or conclusions; duplicate publication; unreliable results or conclusions.

We should note that a single dose of DNMT inhibitor reversed the laser-induced increase in D1 spine density while D2 spine density did not change significantly. Once the synaptic strength of D1 spines is reduced, the inhibitory D2 spines presumably rebalance BLA-DLS circuit leading to suppression of anomalous behavior and perhaps contributing to LTD in D1s.

A similar regulatory interplay of D1 and D2 mediated sub-circuits was found in fear extinction studies, which may point to a generic regulatory/neuroplasticity mechanism across various forms of memory and learning where epigenetic changes play a key regulatory role^62^.

Our results indicate that both the development and reversal of OCD-like behaviors involve neuroplasticity resulting in circuitry changes in BLA-DLS and possibly elsewhere. Particularly, in laser-stimulated mice we observed long-term potentiation of D1s, whereas in RG108 treated laser-stimulated mice we observed normalization of behavior associated with long-term depression of D1s. The observed LTP and LTD through BLA-DLS pathway modulations appear to involve regulatory epigenetic changes. In that context, DNA methylation changes associated with OCD-like behaviors are likely to engage methyl-CpG-binding protein 2 (MeCP2) as one of the regulatory mediators. MeCP2 is a regulatory factor that binds to common DNA methylation site CpG, which in turn affects the expression of multiple genes^63^. MeCP2 has essential maintenance role in mature adult neurons and modulates both synaptic development and function. Loss-of-function mutations of MeCP2 cause neurodevelopmental disorder Rett Syndrome in humans and neurological dysfunction in mice characterized by impaired memory/learning and low synaptic density^64^. The demethylation we induced indirectly by DNMT inhibitor would be expected to have some functional similarities to the loss of MeCP2 as both should counteract the effects of methylation–either via elimination of methyl-CpG sites or via lack of the regulatory factor binding to methyl-CpG, correspondingly. In fact, D1 spine density reduction in DLS that we observed after RG108 administration is consistent with prior findings that the lack of MeCP2 is associated with low synaptic density^65^. This phenomenon is likely to be partly mediated by mTOR pathway that we discussed earlier. A loss-of-function MeCP2 gene mutation leads to reduction in mTOR pathway activity (greater autophagy) and reduced neuronal size in mice^64^.

The article "Amelioration of obsessive-compulsive disorder in three mouse models treated with one epigenetic drug: unraveling the underlying mechanism" was retracted in 2021. Reasons: errors in the materials; errors in the results or conclusions; duplicate publication; unreliable results or conclusions.

Importantly, MeCP2 appears to modulate the inducibility of some of the immediate early genes (IEG) of synaptic plasticity, which was shown specifically in striatum for *junb* and *Arc*^63^. In that context, the effects of methylation and MeCP2 on Arc expression appear particularly relevant because Arc was shown to be involved in complex regulation of various forms of neuroplasticity, including LTP, LTD and synaptic scaling^66,67^. Particularly noteworthy are recent studies showing the capability of Arc protein to transport different payloads, such as RNA, between neighboring dendrites and neurons^68^. Under certain conditions, Arc proteins assemble into carrier particles resembling a viral capsid that can be transported in and out of neurons via endo/exocytosis^68^. The nature of the cargo, co-factor binding and other insufficiently understood variables apparently determine the Arc’s role in each particular type of plasticity. The inter-neural transport mechanism facilitated by Arc is consistent with Hebbian cooperativity characteristic of both LTP and LTD^69^. Epigenetic control of Arc-dependent pathways appears to be a promising avenue of future research.

While epigenetic drugs, and methylating/demethylating agents in particular, appear to hold promise for mental health disorders, there is a potential for significant side-effects. In particular, methylation/demethylation may lead to long-term changes in the activity of oncogenes and conceivably to an increase in the rates of cancer. Further research is needed to identify such risks and find ways to mitigate them. It is likely that different methylating/demethylating agents affect methylation patterns somewhat differently and thus carry different levels and types of risks and benefits. Such differences may be due to DNMT or TET enzyme subtype specificity, involvement of different DNMT-inducing complexes, DNA conformation or sequence specificity and other factors. In fact, some DNMT inhibitors appear to produce anti-cancer effects, presumably by reversing the silencing of tumor suppressor genes^70,71^. Other approaches to reducing the side-effects of epigenetic drugs could include reducing the effective dosage by combining them with relevant non-epigenetic drugs or targeting only specific tissues. For example, the effective dosage of the epigenetic drugs in treating disorders associated with abnormal neuroplasticity, such as OCD or phobias, might be lowered by concurrently administering non-epigenetic neuroplasticity enhancing agents, such as edonerpic maleate^72^. Also, when treating neurological or psychiatric conditions with epigenetic drugs, it should be feasible to preferentially target the nervous system by leveraging the properties of the blood-brain barrier. For example, a small molecule drug, such as RG108, that crosses the blood brain barrier (BBB) may be co-administered with a neutralizing agents, such as an antibody, that does not cross the BBB, potentially leading to effective concentrations only in the CNS. Alternatively, an epigenetic drug that does not cross the BBB could be administered intrathecally, reaching effective concentrations only in the CNS^73^.

The article "Amelioration of obsessive-compulsive disorder in three mouse models treated with one epigenetic drug: unraveling the underlying mechanism" was retracted in 2021. Reasons: errors in the materials; errors in the results or conclusions; duplicate publication; unreliable results or conclusions.

This study has demonstrated the involvement of epigenetic mechanism in the behavioral and circuitry changes associated with the development and reversal of maladaptive habitual behaviors. We focused on the BLA input to the DLS. The BLA modulates the DLS activity via the two opposing pathways of movement stimulation (D1) and movement inhibition (D2), whose anomalies we showed to be associated with OCD-like behaviors. However, similar regulatory circuits and mechanisms appear to be involved in many other brain structures and functions where epigenetic interventions may also have therapeutic potential. Hence better understanding of these mechanisms may lead to new treatments not only for obsessive-compulsive disorder but also many other pathologies characterized by aberrant synaptic plasticity and circuitry dysregulation persisting due to epigenetic changes

## Methods

### Animals

We used 3–6 month old male and female Slitrk5 and SAPAP3 KO mice^34,35^. SAPAP3 mice were used at 3–4 months of age (when they are symptomatic). Because Slitrk5 mice display a protracted disease progression when crossed onto a C57BL/6-SV129 background, they were used at 5–6 months. We used 3–6 month old male and female mice for the WT laser-stimulated mouse model, hemizygously expressing either drd1-tdTomato or drd2-eGFP^74,75^. All mice were housed individually in home cages with 12 h light/dark cycle with food and water ad libitum. All animals in all groups received the same treatment (except for the active agent being investigated, such as an epigenetic drug or laser stimulation). The control and experimental groups underwent the same procedures. The research complied with the National Institutes of Health Guide for Care and Use of Laboratory Animals, and was approved by the Animal Welfare Committee of our institute, NY, USA.

The article "Amelioration of obsessive-compulsive disorder in three mouse models treated with one epigenetic drug: unraveling the underlying mechanism" was retracted in 2021. Reasons: errors in the materials; errors in the results or conclusions; duplicate publication; unreliable results or conclusions.

### Surgeries

For stereotaxic surgery, rats were anesthetized with ketamine and xylazine and secured in a Leica Biosystems stereotaxic apparatus. WT mice received unilateral injections of synapsin-ChR2-GFP-AAV^76^ construct (UPenn vector core) at 2–5 months of age. Stereotaxic injections targeted the BLA (ML −2.99, AP −1.22, DV −4.38). In the same surgery, a mono fiber optic cannula (core diameter 200 μm, outer diameter 245 μm, 0.37 NA, Doric Lenses) was implanted in the dorsolateral striatum (0.6 mm anterior to Bregma, tip depth 2.7 mm below pia surface) and held in place with dental cement. After the implantation surgery, animals were allowed to recover for 5 to 7 days.

### Behavior

Two weeks following surgery, cannula were magnetically coupled to a fiber optic patch cord attached to a 473 nm blue LASER, and placed in a clear Plexiglas cylinder (13 cm diameter). Mice were acclimated to this configuration for 3 days, 20 minutes per day. After acclimation and baseline measurements, the dorsolateral striatum was stimulated by the LASER using 10 ms pulses (3 mW) at 10 Hz for 10 minutes, once daily for 5 days,  based upon previous studies^77^. Control mice received saline injections or sham cannula implants. Mice were videotaped in the Plexiglas cylinder to assess grooming during 3 epochs: (i) 5 minutes before laser stimulation, (ii) during laser stimulation, and (iii) 5 minutes after laser stimulation. Grooming was also assessed for 3 days before the first stimulation, and 1 week following the last LASER stimulation. Total time spent grooming, number and duration of grooming bouts, and body region groomed (head, core or tail) was quantified by observers blind to experimental conditions.

Open field behavior and performance in an elevated plus maze were tested after the stimulation protocol as general measures of locomotion and anxiety-like behavior^78,79^, and analyzed with EthioVision XT software. Data from drd1-tdTomato and drd2-eGFP mice were pooled for behavioral analysis.

### Electrophysiology

The mice were anesthetized with a mixture of ketamine (50 mg/kg) and xylazine (4.5 mg/kg) and perfused transcardially with 5–10 ml ice-cold artificial CSF (ACSF) containing (in mM): 124 NaCl, 3 KCl, 1 CaCl_2_, 1.5 MgCl_2_, 26 NaHCO_3_, 1 NaH_2_PO_4_, and 16.66 glucose, continuously bubbled with carbogen (95% O_2_ and 5% CO_2_). The slices were then transferred to a holding chamber where they were incubated in ACSF containing (in mM) 2 CaCl_2_, 1 MgCl_2_, at 35 °C for 60 min, after which they were stored at room temperature until recording. Identified SPNs were recorded from on a multi-photon system equipped with integrated electrophysiological capabilities. The recording electrode contained (in mM) for current-clamp recording: 135 K-gluconate, 7 KCl, 10 HEPES, 10 Na-phosphocreatine, 4 Mg_2_-ATP, and 0.4 Na-GTP (290–295 mOsm, pH 7.35 with KOH). Voltage-clamp recordings used (in mM): 135 Cs-gluconate, 10 HEPES, 10 Naphosphocreatine, 4 Mg_2_-ATP, and 0.4 Na-GTP (290–295 mOsm, pH 7.35 with CsOH) and red fluorescent anatomical dye Alexa 568 (50 μM) (Invitrogen). ChR2 stimulation of BLA terminals in the DLS were evoked by stimulating the DLS with two laser pulses 400 μm away from the neurons. Excitatory postsynaptic currents (EPSCs) were recorded from a projection neuron in the DLS in response to optogenetic paired-pulse stimulation (1 ms) with an interval of 100 ms. The averaged paired-pulse ratio of the amplitudes (PPR = EPSC2/EPSC1) were calculated after recording.

The article "Amelioration of obsessive-compulsive disorder in three mouse models treated with one epigenetic drug: unraveling the underlying mechanism" was retracted in 2021. Reasons: errors in the materials; errors in the results or conclusions; duplicate publication; unreliable results or conclusions.

In order to detect changes in NMDA/AMPA ratios, we recorded in voltage clamped SPNs BLA input laser stimulation evoked AMPA currents at −70 mV, and NMDA currents at +40 mV^80,81^.

For spine density studies, high magnification z-series images (0.2 μm steps, 5x digital zoom) were taken through two distal (>100 μm from soma) and proximal (60 μm from soma) dendritic areas. The distance from soma was measured by a straight line drawn from the site of stimulation to the origin of the dendrite at the soma. The images were de-convoluted using AutoQuant X2 (Media Cybernetics) and for spine density analysis we used neuron studio64^82^.

Low magnification z-series images (1 μm steps, 1x digital zoom) were taken through the depth of the entire recorded neuron.

### Drugs

RG108 (Sigma) was dissolved in 10% DMSO and sterile saline and injected subcutaneously at 0.8 mg/kg dosage. Sodium butyrate (NaB, Sigma) was dissolved in sterile saline and injected subcutaneously at 1.2 mg/kg dosage.

### DNA Methylation Assay

This DNA methylation assay was performed as published by^21^. Detection of un-methylated *PP1* DNA was performed using the following primer^21^: Forward (5′-GAGGAGAGTTTGGTGTTTATAAGATGGT-3′) and reverse (5′-TCCTCCAAAAACTCAACTCAAACAA-3′). Detection of methylated *PP1* DNA was performed using the following primer^21^: Forward (5′-GGAGAGTTTGGTGTTTATAAGATGGC-3′) and reverse (5′-CGAA AACTCGACTCGAA CGA-3′). PCRs were performed in a StepOnePlus real-time PCR system (ThermoFisher). To further verify specificity of the final product, 5 μl of the amplified products were analyzed by electrophoresis on a 2% agarose gel stained with ethidium bromide and visualized under UV light. Quantitative PCR was run three times with each sample. For every quantitative PCR, samples were assayed in triplicate and the Ct value for each sample was chosen in the linear range. Samples were normalized to a control unstimulated and untreated WT sample, and the comparative Ct method was used to calculate differences in gene expression between samples (log-2-fold-change).

The article "Amelioration of obsessive-compulsive disorder in three mouse models treated with one epigenetic drug: unraveling the underlying mechanism" was retracted in 2021. Reasons: errors in the materials; errors in the results or conclusions; duplicate publication; unreliable results or conclusions.

### Statistical analysis

All data were presented as the mean ± standard error. All statistics were performed using GraphPad Prism 5.0b. Comparison between two groups was evaluated by an unpaired Student’s t-test. Differences between treatment groups were evaluated using one-way or two-way ANOVA with Tukey post hoc comparison tests. Statistical significance was defined as p < 0.05.

## Data Availability

The data that support the findings of this study are available from the corresponding author (C.C.), upon reasonable request.
